The article "Effectiveness of option B highly active antiretroviral therapy (HAART) prevention of mother-to-child transmission (PMTCT) in pregnant HIV women" was retracted in 2014. Reasons: ethical violations by an author; no approval from the institution.

# Effectiveness of option B highly active antiretroviral therapy (HAART) prevention of mother-to-child transmission (PMTCT) in pregnant HIV women

**DOI:** 10.1186/1756-0500-7-52

**Published:** 2014-01-21

**Authors:** Erastus K Ngemu, Christopher Khayeka-Wandabwa, Eliningaya J Kweka, Joseph K Choge, Edward Anino, Elijah Oyoo-Okoth

**Affiliations:** 1 School of Science, Department of Biochemistry, University of Eldoret, PO Box 1125, Eldoret, Kenya; 2 Institute of Tropical Medicine and Infectious Diseases (ITROMID), Jomo Kenyatta University of Agriculture and Technology (JKUAT), Nairobi, Kenya; 3 Tropical Pesticides Research Institute, Division of Livestock and Human Diseases Vector Control, Mosquito Section, Ngaramtoni, Off Nairobi road, PO Box 3024, Arusha, Tanzania; 4 School of Health Sciences, University of Eastern Africa, Baraton, PO Box 2500-30100, Eldoret, Kenya; 5 School Natural Resources and Environmental Studies, Karatina University, PO Box 1957-10101, Karatina, Kenya

**Keywords:** Antiretroviral, CD4 counts, Early Infant Diagnosis, Highly Active Antiretroviral Therapy (HAART), Mother-To-Child Transmission (MTCT), Prevention of Mother-To-Child Transmission (PMTCT)

## Abstract

**Background:**

Ensuring that no baby is born with HIV is an essential step towards achieving an AIDS-free generation. To achieve this, strategies that decouple links between childbirth and HIV transmission are necessary. Traditional forms of prevention of mother-to-child transmission of HIV (PMTCT), has been recommended. Recognizing the importance and challenges of combination of methods to achieve rapid PMTCT, the World Health Organization (WHO) recommended option B Highly Active Antiretroviral Therapy (HAART) for all HIV-positive pregnant women. This study aimed to evaluate the effectiveness of the HAART in PMTCT. A cohort of HIV-infected pregnant women in Kenya were obtained from the DREAM Center, Nairobi. The study participants underwent adherence counselling and Option B of HAART [Nevirapine(NVP) + Lamivudine + Zidovudine] at the fourth week of gestation followed by an intravenous NVP administration intrapartum and postpartum NVP syrup to the respective infants for six weeks. Absolute pre-HAART and post-HAART CD4 counts and viral loads counts were determined. Comparison of the CD4 counts and viral loads before and after administration of HAART were done using Wilcoxon’s Matched Pairs Signed-Ranks Test.

**Findings:**

The mean absolute CD4 cell counts in mothers after administration of HAART was significantly higher (Z = 15.664, p < 0.001) than before the administration of HAART). Also the viral load of the mothers significantly (Z = 11.324, p < 0.001) reduced following HAART treatment. Following the HAART administration in mothers, up to 90% of children were confirmed to be HIV negative.

**Conclusion:**

Administration of HAART to mothers and children demonstrated an effective mechanism of PMTCT. However, other aspects of HAART such as adherence, costs, mothers behaviour during HAART, and the child feeding programme during the therapy should further be evaluated and ascertained how they can affect the overall efficacy of option B HAART in PMTCT.

## Findings

Socio-demographic characteristics of the 50 individual mothers selected for this study is provided in Table 1. Most of the study population were aged 23 to 32 years and were mainly married. Majority of the women (56%) had secondary level of education. Over 68% of the women sampled reported that they were self-employed with another 28% being unemployed.

**Table 1:** Characteristics of the study subjects (n = 50)

**Characteristics**	**Frequency**	**Percent**
**Age (in years)**		
18–22	4	8%
23–27	17	34%
28–32	22	44%
33–37	7	14%
**Marital status**		
Married	24	48%
Single	15	30%
Divorced	3	6%
Widowed	8	16%
**Occupation**		
Self employed	34	68%
Civil servant	2	4%
No form of employment	14	28%
**Education level**		
None	3	6%
Some primary/primary	15	30%
Some secondary/secondary	28	56%
Middle level college/University	4	8%

Information on the absolute CD4 counts of mothers before and after administration of HAART during the study is shown in Figure 1. The mean (± SEM) absolute CD4 cell counts in mothers after administration of HAART (496.38 ± 16.32 counts/ml) was significantly higher (Z = -15.664, p = 0.00003) than before the administration of HAART (435.86 ± 17.32 counts/ml).

**Figure 1:** Mean (±SEM) absolute CD4 cell counts before and 6 months after administration of option B HAART to the mothers (n = 50).

We also determined changes in the viral load in mothers before and 6 months after the administration of HAART therapy and similar parameter in children 6 weeks after birth under HAART treatment (Figure 2). Viral load of the mothers before HAART treatment was obviously high for most the study subjects (17,555 ± 1,458 copies/ml). However, there was a significant (Z = 11.324, p = 0.00008) reduction in the viral load of the mothers after HAART treatment (11234 ± 965 copies/ml).

**Figure 2:** Mean viral load counts before and 6 months after administration of option B HAART to the mothers (n = 50) and in children 6 weeks after HAART (n = 50).

We also tested the PMTCT regimen effectiveness using the number of 6 weeks children that were HIV-free. Based on a sample of 50 children, our result indicated that, 45 children had viral load less than 50 copies/ml 6 weeks after birth indicating 90% effectiveness of Option B highly active antiretroviral therapy PMTC in children in the current study.

### Background

Continuing expansion of the HIV/AIDS pandemic among women has been recognized as an exceptional challenge to global maternal health. Each year, around 1.5 million women living with HIV become pregnant and deliver [1]. About 90% these women live in Sub Saharan Africa (SSA) where comprehensive health services and HIV medication regimens are limited [2]. In absence of interventions, the HIV-infected mother has a 15–45% chance of transmitting the virus to her newborn during her pregnancy or birth, or via breast milk [1]. A worrying trend indicates that 90% of new infections in children are due to mother-to-child transmission (MTCT). In 2011, around 330,000 children living in SSA under the age of 15 became infected with HIV via MTCT pathway [3]. Thus prevention of MTCT (PMTCT) is critical in curbing the spread of new HIV infections.

The global community has committed itself to accelerate progress for the PMTCT initiative to eliminate new paediatric HIV infections by 2015 and improve maternal, newborn and child survival in the context of HIV. PMTCT advocated by UNAIDS entail (1) keeping women of reproductive age and their partners HIV-negative through reproductive health and HIV prevention services, (2) avoiding unwanted pregnancies among HIV-infected women and women at risk of HIV, through family planning and HIV testing and counselling services and (3) ensuring HIV testing of pregnant women and timely access to effective antiretroviral therapy, both for the health of HIV-infected mothers and for PMTCT, during pregnancy, delivery and breastfeeding [3]. Adherence to these practices is highly variable with better results obtained in developed countries than in the developing countries.

Mothers partaking PMTCT have reduced the risk of MTCT to less than 5% [4]. In the developed world where PMTCT through access to comprehensive testing, effective voluntary testing and counseling services and treatment, the rate of MTCT of HIV is less than 2% [5,6]. Globally, since 1995, more than 350,000 children annually have avoided HIV infection due to these interventions [7]. Not surprisingly, inadequate continuum of care, magnitude of PMTCT and associated services including HIV testing and counseling and ARV prophylaxis are still very low in developing countries [8,9]. A UNAIDS report estimated only 5% of HIV-infected women accessed PMTCT interventions in a surveillance of 30 African countries with the highest HIV prevalence [3]; a huge shortfall from the UN target of 80% by 2010 (http://www.unaids.org/en/KnowledgeCentre/HIVData/GlobalReport). Continued research that tends to accelerate PMTCT appears effective in eliminating new HIV infections among children. Against the context of evolving evidence, constant revision of national PMTCT guidelines and policy choices may be vital.

In PMTCT, consortia of antiretroviral drugs (known as highly active antiretroviral therapy HAART) that decouple links between childbirth and HIV transmission are adopted. The use of multiple drugs, often referred to as a “cocktail”, serve as powerful defenses against the ways in which the HIV virus attacks the human body. Although these drugs are not able to rid the body of HIV, they can significantly delay the onset of AIDS and potentially slow down the replication of HIV lowering the viral load in the mother’s body and hence reducing the chances of HIV transmission. The current WHO recommended regimen is as follows: where the pregnant woman does not yet need to start ART for therapeutic reasons, she should start Zidovudine (AZT) from 28 weeks or as soon as possible thereafter, be provided with single-dose Nevirapine (NVP) when entering labour, and be given AZT + 3TC for one week following delivery. Meanwhile, whether the mother was on the above or standard ART, the child should be given single dose NVP immediately after delivery and daily AZT until one week old (http://www.who.int/entity/hiv/pub/guidelines/pmtctguidelines3.pdf). Complementary measures that may also be used include caesarean section and formula feeding; in some settings, the combination of providing all these measures has been used with variable success [10]. However, HAART is still often described as having miraculous effects. Not surprisingly, proponents of these drugs are less anxious to discuss the times when the drugs simply do not seem to do what they are supposed to in terms of its effectiveness. The aim of current study was therefore to evaluate the effectiveness of HAART in reducing cases of MTCT of HIV in resource-limited settings in Kenya.

Kenya is characterized by high prevalence of HIV. The Kenya National AIDS/STI Control Programme (NASCOP) estimates that 6.3% of pregnant women are living with HIV/AIDS in Kenya [2]. Similar to situations in other developing countries, a high number of people living with HIV/AIDS are within the reproductive age bracket (15–49 years old) and are mainly women. In the absence of PMTCT services, estimated 60–90% of MTCT risks is a reality [11]. This was gradually recognized and subsequently the Ministry of Health in Kenya, recently recommended the use of HAART in the country. However, there is still lack of information on the effectiveness of HAART in PMTCT.

## Methods

During the period between November 2009 and January 2011, we carried a cross-sectional study at the Daughters of Charity of St. Vincent De Paul DREAM Centre in Nairobi, Kenya. The facility incorporates a fully functional Voluntary Counselling and Testing Centre (VCT) and a diagnostic laboratory for conducting haematological and serological assays. The centre provides both comprehensive and holistic care to the approximately 2000 people living with HIV/AIDS (inclusive of men, women and children) under their care. In the centre, diagnostics, nutritional support, health education and treatment of opportunistic co-infections of HIV/AIDS are offered at no charge.

During the study, 50 pregnant HIV positive pregnant women who visited the centre to access both pre-natal and post-natal care services were selected. The HIV positive status of the pregnant women were either confirmed at the centre or pre-tested during previous ante-natal visits. The subjects were provided Option B HAART as per 2010 WHO PMTCT guidelines WHO (2010). During the six month treatment. Three ARV drugs namely NVP, + Lamivudine and Zidovudine were administered to each of the study participants starting at fourth week of gestation, followed by adherence counselling. After birth, an intravenous NVP administration intrapartum and postpartum NVP syrup was also administered to infants for six weeks [4]. Where available, previous medical records helped to provide baseline information of the participants before undertaking actual clinical tests. The study period lasted for over one year spanning right from the onset of the pre-natal administration of HAART drugs, lasting through the 2^nd^ and 3^rd^ trimesters of pregnancy, delivery and culminated in the assessment of the post-HAART outcomes for the paediatric populations. The results considered were for those pregnant women who adhered to the HIV chemoprophylaxis agents (HAART) administered to them for the whole duration of the PMTCT programme which lasted for a period not less than six months. Consideration in the patient’s records was information such as date of HIV diagnosis and CD4 count assays if any, HIV viral load, previous illness and treatment received before. Women who did not meet the criteria were excluded from the study. All patients who met the criteria and were willing to participate in the study and gave informed consent were included.

On testing positive, the women had their pre-HAART viral load (copies/ml) and CD4 absolute counts determined. These women were then placed on an Option B HAART regimen to act as a chemoprophylaxis for the HIV. They were continually monitored for adherence to the HAART regimen, manifestations of side effects and opportunistic infections through clinical recaps. Pre-HAART and post-HAART CD4 absolute counts were established using a BD Biosciences FACS Calibur flow cytometer. The study participants were appropriately advised to undergo elective caesarean method of delivery as is the conventional practice in PMTCT programmes. Upon successful delivery, the post-HAART serum viral loads of all the neonates born to the study participants were monitored postpartum (DNA-PCR conducted at six weeks after birth). Changes in the viral load in mothers before and after the administration of HAART therapy were also determined. All these parameters were employed as indicators for the effectiveness of the HAART regime in the PMTCT programme. Follow-up was also made as a routine of the centre to monitor compliance to the ARVs and that the babies were fed as advised so as to avoid the risk of MTCT of HIV during lactation and weaning periods through a consistent recap on clinical visits [11,12]. The response to ARVs as well as the occurrence of any opportunistic infections, such as tuberculosis, was also monitored. The sample of 50 for the study was calculated using the Java Applets for power and sample size software [13]. Hence to meet the estimated numbers of 50 patients, 63 were screened, considering likely losses during follow-up. All respective ethical clearance from DREAM centre was adhered to and considerations as pertaining confidentiality, beneficence and justice were followed and all the data collected was treated with anonymity. Two outcomes of interest were considered to evaluate PMTCT regimen effectiveness: the number of 6 weeks children that were HIV-free i.e. viral load less than 50 copies/ml and changes in viral load and CD4 counts in mothers.

All statistical analyses were performed with a version of STATISTICA 10.0 statistical packages. Comparison of the CD4 counts and viral loads before and after administration of HAART were done using Wilcoxon’s Matched Pairs Signed-Ranks Test as count data take discreet variables. All analysed results were declared significant at p < 0.05.

The study obtained ethical clearance from the Moi University Institutional Research and Ethics Committee (IREC), (Formal approval no.: FAN: IREC 000301). Supportive letter was obtained from the district health office before data collection, and written informed consent was obtained from voluntary participants and parents or guardians for children during data collection.

## Discussion

Although in developed countries HIV incidence are low [14], most new cases continue to emerge from developing nations [3] hence more research focus of HIV research in these areas. Unfortunately, the high incidence is not likely to change in the foreseeable future because: (1) HIV-prevention strategies are only partly effective and remain severely underused [15-17]; (2) a preventive vaccine remains elusive [18] and (3) current treatment strategies cannot eradicate HIV infection [19-23]. Therefore, management regimen of HIV infections still relies on the effective use of prevention of occurrence or spread of the HIV virus. It is well recognized that MTCT is one of the ways in which HIV virus is perpetuated from one generation to another. Containance of the HIV infection has therefore continued to focus on PMTCT. Accordingly, WHO recommends option B, a triple ARV prophylaxis in HIV infected pregnant women in attempt to enhance PMTCT programmes [2,24]. In this programme, triple ARV therapy is continued postpartum without interruption irrespective of CD4 count, WHO clinical stage or breastfeeding status [8,25-27]. Yet, little research output is available on the use of option B HAART. Therefore the aim of the current study was to determine the effectiveness of Option B HAART in PMTCT in Kenya, one of the developing countries. We ensured effective administration and adherence to Option B HAART regimen among the study subjects by continous counselling, comprehensive education advise before commencement of treatement programme and nutrional support thus minize experimental error.

During the study, the absolute CD4 cell counts in mothers after administration of HAART was established to be significantly higher than before the administration of HAART. This suggests an increased CD4 counts following Option B HAART therapy. This observed increase of the CD4 counts could be due to the ability of HAART to reduce HIV-1-RNA plasma concentrations predictably to undetectable concentrations in most treated patients as was previously shown [28]. Moreover, the international guidelines have uniformly recognized that sustained complete suppression of HIV-1-RNA is needed to achieve a steady increase in CD4- T-lymphocyte (CD4) cell count as well as a beneficial clinical response, and to avoid the emergence of drug resistant HIV mutants [29]. Furthermore, the use of HAART has been reported to leads to a marked reduction in HIV-1 RNA concentrations in both the female genital tract and in semen [30,31], which may result in a reduction of the risk of viral transmission during sexual intercourse.

The relationship between viral load and HIV infection in heterosexual couples is clearly understood. For instance, it has been reported that viral load is the main predictor of the risk of transmission of HIV, in heterosexual couples and that transmission is rare in those with plasma HIV-1-RNA concentrations of less than 1500 copies per mL [32]. Similarly, Tovanabutra and others showed a dose–response effect between viral load and risk of HIV transmission within sero-discordant heterosexual couples [33]. No cases of HIV transmission were seen when the index case’s plasma HIV-1-RNA was less than 1100 copies per mL in the same study. As yet, the threshold viral load for transmission of MTC is not clearly known. In this study, we established that the viral load of the mothers reduced by 36% following HAART treatment, suggesting a higher probability of reduced vertical transmission of HIV that may have an impact on the overall levels of MTC. A study in Taiwan, provided a compelling evidence about the effect of HAART on HIV transmission [34]. The study showed a 53% reduction in new positive HIV tests after the introduction of free access to HAART. In British Columbia, Canada, new HIV infections fell between 1995 and 1998 after the introduction of HAART by about 50%, and have remained unchanged to the present [22]. Further ecological evidence of an effect of HAART on HIV transmission can be derived from a detailed review of the UNAIDS statistics [25,26]. In 2005, about 38,600,000 people were estimated to be living with HIV or AIDS worldwide, with more than 4,000,000 new HIV infections and 2,800,000 AIDS-related deaths in that year. The numbers of people living with HIV, numbers of new HIV infections, and the ratio of new HIV infections per 100 people living with HIV in 2005 show clear spatial difference by regions, which correlated inversely with regional availability of HAART. We therefore hypothesize in the current study that the reduced viral load in mothers may result in increased PMTCT.

Evidence of the effect of HAART on the prevention of HIV transmission was evidently derived from the current study. We established that up to 90% of children were confirmed to be HIV negative with less than 50 copies/ml of viral load following HAART therapy in which the mother were provided with the combination therapy. This indicates 10% MTCT. We provided combined antepartum, intrapartum, and infant antiretroviral prophylaxis to the children which can potentially reduce perinatal transmission by lowering maternal antepartum viral load and pre- and post-exposure prophylaxis of the infant. The present study findings are superior to previous results in which lower percent reduction in HIV prevalence was reported when only anti-retrovirals (i.e. zidovudine alone) were the most preffered tool in managing vertical transmission [35]. The present PMTCT findings are lower than in the developed countries (about 1%) due to the combination of widespread access to anti-retroviral therapy (ART), elective caesarean sections (ECS), safe formula feed and access to quality medical services that conspicously lack in developing countries [36]. However the current effectiveness level of 10% was comparatively higher than the average rate in most of the countries in the developed world, which is estimated at about 1% [3]. Even before the HAART era, the key role of maternal plasma HIV-1-RNA concentrations in HIV transmission had been suspected [34,37]. Subsequently, clinical trials have shown that reducing the mother’s plasma HIV-1-RNA concentration with HAART dramatically reduces mother-to-child transmission of HIV [38,39].

Although Option B HAART proved efficacious in PMTCT, some limitations may have to be pointed out. The number of transmitted cases from MTC might not be exactly proportional to prevalence of HIV infection, because a limited number of individuals with very high viral load could contribute a disproportionate number of transmission events. Also, HAART might not be the only factors that contribute to reduced transmission in the study area since, traditional herbal medicine are also rampantly used in the areas where our study subjects came from. We must stress that we do not see Option B HAART as a replacement for strengthening of the PMTCT, but rather as an essential part of it. The role of counseling, comprehensive advice before commencement of treatment programme and nutritional support are also adviced to enhance full adherence to the programme. In resource poor areas, many mothers do not have access to the clean water and fuel that make replacement feeding feasible and safe a factor that was attested at DREAM Centre based on the nutritional support. HAART prophylaxis and infant feeding counseling and education must be made available and/or emphasized as part of the standard of pre-natal and post-natal care for pregnant women who are diagnosed HIV-positive.

## Conclusion

The present approach to the management of HIV/AIDS which involve the use of ARVs alone have clearly been found not sustainable, and the status quo no longer acceptable if we hope to control the continued growth of the HIV global pandemic. A prevention-centred approach in the present study elucidated that the use of Option B HAART ensured up to 90% effectiveness in the PMTC. This implies that MTCT rate with administration of HAART is as low as 10%. We therefore recommend the combination antiretroviral regimens containing at least three drugs (i.e. Option B HAART) as well as comprehensive advice/counseling before commencement of treatment programme and nutritional support are also advised to enhance full adherence to the programme and for prevention of prenatal HIV transmission, which should be offered to all HIV positive pregnant women. Other limitations to the use of HAART in PMTCT of HIV also need to be studied and reduced to enhance its maximum utilization in many developing countries where the MTCT is currently highly prevalent.

## Competing interests

The authors declare that they have no competing interests.

## Authors’ contributions

EKN, EJK, CK-W and JKC conceived and designed the study; EKN, CK-W and JKC collected data; EA provided logistical support during research design and data collection. CK-W, EO-O, EKN, EJK and JKC participated in drafting and revising the manuscript. EO-O analyzed the data. All authors approved the final manuscript.
